RETRACTED

# Effect of Vegetable Waste on Growth Performance and Hematology of Broiler Chicks

**DOI:** 10.1155/2022/4855584

**Published:** 2022-10-10

**Authors:** Muhammad Shahid Nisar, Anjum Zahra, Muhammad Fahad Iqbal, Muhammad Amjad Bashir, Riffat Yasin, Khizar Samiullah, Irum Aziz, Sidra Saeed, Abdulrahman Alasmari, Fahmy G. Elsaid, Ali A. Shati, Mohammed A. Al-Kahtani, Farwa Naseem, Maryam Fatima, Faraz Ahmed

**Affiliations:** ^1^Department of Plant Protection, Ghazi University D. G. Khan, Pakistan; ^2^DHQ teaching hospital Dera Ghazi Khan Punjab, Pakistan; ^3^Avicenna medical college Lahore Punjab, Pakistan; ^4^Faculty of Veterinary and Animal Sciences, MNSUA, Multan, Pakistan; ^5^Department of Plant Breeding & Genetics, Ghazi University D. G. Khan, Pakistan; ^6^Department of Zoology, Ghazi University D. G. Khan, Pakistan; ^7^Department of Biology, Faculty of Sciences, University of Tabuk, Tabuk, Saudi Arabia; ^8^Biology Department, Science College, King Khalid University, Abha, Saudi Arabia; ^9^Zoology Department, Faculty of Science, Mansoura University, Mansoura, Egypt; ^10^WMO RHD (Rural Health Dispensary), Badduke, Lahore, Punjab, Pakistan; ^11^WMO at RHD kmahan, Lahore, Punjab, Pakistan; ^12^Basic Health Unit Faizabad tehsil Depalpur District Okara Punjab, Pakistan

## Abstract

Vegetable waste (spinach, potato, and cauliflower) is a rich and natural source of nutrients, potentially good for supplying minerals, essential amino acids, and antioxidants to the birds. Relatively, its cost very low, easily to accessible, easily process & pose little risk of illness. The aim of present study was to evaluate the effect of vegetable waste (VW) as feed supplement on growth performance and hematology of broiler chicks. For this purpose, a total of 200 (4 days old) vaccinated chicks were acquired from a commercial hatchery Multan which was acclimated for three weeks (21 days) on basal starter feed after that 25-day-old chicks with uniform body weight were allocated according to a CRD (completely randomized design) into four dietary treatments with three replicates of each contained 15 chicks in 12 pens. In dietary treatments, chicks were feed with basal feed (BF) and supplemented feed with vegetable waste (VW) of spinach, potato, and cauliflower. For this purpose, the dietary treatments included control treatment (*T*_1_) (100% BF+0% VW) and other dietary treatments (*T*_2_) (75% BF+25% VW), (*T*_3_) (50% BF+50% VW), and (*T*_4_) (25% BF+75% VW). The body weight, feed intake, food conversion ratio (FCR), and mortality were checked on weekly and daily basis. For hematology analysis, after the 1st experimental week (25-day-old chicks) and the last 5th experimental week (56-day-old chicks), the samples of blood were gathered from the wing's veins of two birds from each treatment in random way. At the end of five weeks (35 days), birds with uniform average body weight were selected per treatment with three replicates (2 bird/replicate) and then were manually slaughtered according to the Halal method to analyze the weight of internal body organs of broilers by physical and statistical analysis (ANOVA). There was no significant effect (*P* > 0.05) on feed intake and FCR among all the dietary treatments. But in average, body weight and BWG were higher in treatment (*T*_2_) (*P* < 0.01) than all other dietary treatments (*T*_3_) and (*T*_4_) and control treatment (*T*_1_). The blood constituents in this study showed that broilers in control treatment (*T*_1_) and other dietary treatments (*T*_2_), (*T*_3_), and (*T*_4_) fed on different doses were significantly (*P* < 0.01) different from each other. The week 5 (*W*_5_) shows higher values of blood constituents (*P* < 0.01) than week 1 (*W*_1_). The carcass yield of the chicks fed on different doses showed that they were significantly different (*P* < 0.01) among the dietary treatments. The VW inclusion 0%, 25%, 50%, and 75% had positive effect on blood constituents and carcass yield of the broiler chicks; they were significantly (*P* < 0.01) different among the treatments.

RETRACTED

## 1. Introduction

A broiler is any chicken (*Gallus gallus domesticus*) that especially for meat production is raised and bred. In comparison with beef cattle, sheep meat, and pig meat, the broiler chicks due to its less expensive and highly availability have shown an increasing trend across the world. Great flavor, tenderness, and the juiciness are the qualities of the broiler chicken due to its subcutaneous and marbling fat content in the meat and skin which makes the chicken taste more delicious when processed [1]. Broiler meats demonstrate as a functional food with more levels of natural antioxidants [2]. With the sorts of business interests, the poultry industry has become a distinct industry such as egg production, broiler production, hatchery, and poultry equipment businesses and feed mills springing up [3]. The fast growth performance of broilers supports the FCR (feed conversion rations), but users usually accuse about bad juicy nature and aroma of poultry meat. The meat quality improved and the growth rate slows down the commercial broilers by supplementing the vegetable waste (VW). So, the VW supply only maintains their requirements [4].

Across the world, by the change in living way of the society they are becoming much serious and worried about their health performance so, that the need of the people increases for useful and pure functional feeds. So, the meat of broiler is testified as functional food due to more level of natural antioxidants ([5] & Hakim et al., 2022). Food waste (FW) can be avoided around the food supply chain. Avoidable waste food normally thrown out in the land-fills. Food waste if processed and utilized in the right way may consist of high nutrients and energy. The proper processing procedure of green vegetables produced extremely waste material or byproduct, whichever incorporate about 25-30 percent of the whole waste [6]. Consequently, appropriate and organized handlings of food waste (FW) not only produce useful and energetic products but also minimize the crush on the environment [7]. Vegetable wastes are easy to access, found everywhere, and also have high source of nutrients for the broilers to increase body weight, have good meat quality, and provide antioxidant stress to broilers [8]. The broilers which feed on vegetables produce juicy, cholesterol-free, and tenderness meat have highly demanding properties [8].

RETRACTED

Supplemented vegetables to the commercial broilers slow down broilers' growth rate to improve and provide taste in meat quality and supply at low cost to the producers [4]. Spinach has useful constituents in a modern crop with rich nutritional and biological values. Spinach is an excellent supply of nutrients such as manganese, iron, zinc, and magnesium. Spinach also contains little amount of vitamins, like vitamin A, K, E, and C, thiamine (B1), riboflavin (B2), pyridoxine (B6), and foliate. Spinach on dry basis is an excellent source of protein, minerals, iron, and vitamins especially vitamin A, B1, B2, and C [9]. The spinach as a leafy vegetable can dry, handle, and preserve more easily in powder form [10]. The little amount of spinach use as supplemented feed to the chicks did not enhance and better the nutritional rate of the meat but also improved the color quality and taste of the meat [11]. Potatoes are a primary food of many families and potatoes are a versatile root vegetable. Potatoes are low costly and easily grow vegetable which consist variety of nutrients. Due to their carbohydrate level and protein composition, the potatoes are considered as rich source of nutrients. Potatoes are substitute of corn [12]. As compared to the remaining apart of potato (potato tuber), the sweet potato peel contains minerals, large amount of proteins, and other noncarbohydrate compounds [13].

Cauliflower is rich in minerals and lower in calories so, that cauliflower is acceded a vigor food for the chicks. Actually, cauliflower contain approximately every minerals including calcium, iron, vitamin B-6, and vitamin C which feed to chicks as supplement feed become them healthy [14]. The inclusion of SPRM (sweet potato (*Ipomoea batata*) root meal) feed consisted of about 5 percent that was good & guide WG (weight gain), consumption of diet & had not pre contagion ability of initial broiler chickens, not interrupt with process of hematological & so that it was selected for optimum broiler starter production conducted by [15]. The average of vegetable waste used had a substantial impact (p0.05) on live weight, FCR, AMEn, and metabolic crude fiber digestibility, as well as a very massive effect (p0.01) on feed intake, nitrogen retention, and metabolic nutrient digestibility conducted by Fitasari et al. [16]. The powder of spinach impacted flesh color, but not thio-barbituric acid reaction substances or lutenin deposition conducted by [17]. Broilers fed on cauliflower waste as supplemented diets then the feed conversion efficiency increased with minimum cost. Thus, supplemented diet as cauliflower waste to broilers up to 50% level is mostly useful investigated by Kamlesh and Saraswat [18].

RETRACTED

## 2. Materials and Methods

### 2.1. Experimental Site

To investigate the combine effect of vegetable waste like potato, spinach, and cauliflower on the growth and blood hematology of broilers, the experiment was conducted at government poultry farm (Shed) nearby circuit house D. G Khan.

### 2.2. Collection of Samples

Three different vegetables (potato, spinach, and cauliflower) were selected as feed supplement. For the preparation of supplemented feed, the vegetable waste was collected from the local markets, restaurants, and homes at D. G Khan.

### 2.3. Feed Preparation

Vegetable (potato, spinach, and cauliflower) wastes were sliced and dried under the shade to prevent the loss of volatile nutrients. During the drying process, vegetable waste was covered by a fine mesh to keep them clean from dusts. Moreover, regular turning of vegetable waste was done to prevent the possible growth of molds. The air-dried vegetables were crushed in grinder in the form of fine granular powder or granules. The crushed vegetable waste was packed in bags of 100 kg capacity and used for further experimentation.

After that, measured amount of crushed vegetable waste and basal diet (wheat, rice, and millet) was mixed approximately for feeding purpose. So, the measured amount of feed was packed in plastic bags.

### 2.4. Ingredients of the Experimental Diets

The dietary ingredients used in this experiment were wheat, rice, millet, and the three selected vegetable (cauliflower, spinach, and potato) waste. The wheat, rice, and millet were used as basal diet. The vegetable wastes (spinach, cauliflower, and potato) were used as experimental diets with different percentages.

RETRACTED

### 2.5. Experimental Design

The experiment was conducted in CRD (completely randomize design) composed of four (4) dietary treatments replicated thrice. Fifteen chicks were present in each treatment. Treatment (*T*_1_) was considered as untreated controls which were fed only with basal feed (wheat, rice, and millet). The other treatments (T2), (T3), and (T4) were supplemented with vegetable waste (spinach, potato, and cauliflower) along with basal feed at different percentages. Percentage of different feed supplements in all the treatments including control is given in Table 1.

### 2.6. Procurement and Management of Experimental Chicks

Two hundred (*n* = 200) four-day-old broiler chicks were purchased from commercial Multan hatchery. Vaccination was given against main poultry diseases as viral and bacterial diseases accordant to scale granted by Multan hatchery from where the broiler chicks were purchased. The vaccines against the diseases were received from D. G Khan veterinary institute. The broiler chicks were received with standard veterinary training and according to the completed medical care. Their initial weight was measured by weighing machine. At the experimental site, the chicks were raised for three weeks (21 days) in a brooding pen and during that time they were fed starter diets. At the completion of acclimation period (brooding period), twenty-five-day (25) old, one hundred eighty (*n* = 180) chicks with uniform body weight were randomly transferred into experimental pens. Areas given to each group were equal. Each wood mad pen had a 3^∗^4-meter length and was designed to hold 15 chickens, as well as with drinkers and feeders. There were four treatments including one control treatment each with three replicates. Floor bedding was covered with plastic sheets. At a height of around 5 cm, the litters of wood shavings or rice husk were utilized. Those litters were dried completely.

All experimental pens, feeders, and drinkers were cleaned and formalin sterilized firstly. All of the birds were kept in the same circumstances (lighting, temperature, ventilation systems, and moisture content). The average temperature of the experimental setup was 35-37°C. Twenty-four hour lightening system was available according to their need. The feeding trial was carried out from the 3rd to 8th week of age, and therefore, for 5 weeks, each of the four treatments of birds was fed with one of the dietary treatments. Throughout the trial, clean and fresh water was available at all times. The study was carried out for five weeks. Mortality was recorded when it occurred. The vaccination was given at 14th, 21st, and 28th day of the experimental period. Initial and weekly body weight was measured for growth performance. The FCR (feed conversion efficiency) was recorded. Blood samples were taken two times during experimental periods to check the blood status of broiler chicks. Organs' weights were measured after dissection at the end of experimental period for carcass yield.

RETRACTED

### 2.7. Data Calculation and Analysis

Data were collected on daily basis and on weekly basis. On daily basis, feed consumption and feed repulsion were recorded. Each group's body weight and feed intake were monitored on a weekly basis.

The following analyses were performed to check the impact of VW (vegetable waste) on growth performance and hematology of broiler chicks.

- Growth performance analysis
- Blood constituents analysis
- Statistical analysis

### 2.8. Growth Performance Analysis

During the experimental trail, the broiler chicks had been fed on a replica basis according to the applied feed scale, with a measured amount of diet provided each day between 8 : 00 am and 16 : 00 am. Before offering and weighing feed, the rejected feed always was gathered every next morning. The amount of feed consumed was then calculated by subtracting the repelled feed from the applied feed. The weight of body was measured at the start of the trial (called the initial weight) and subsequently on a weekly basis before feeding between 7 and 8 a.m. The ultimate body weight gain was observed by taking a weight of body at the ending of the experimental time period. After that, the total BWG (body weight gain) was determined by subtracting the starter and ended body weights. Mortality was calculated on daily bases. Total feed consumption and total BWG (body weight gain) were used to determine the FCR.

The feed conversion ratios (FCR) were measured by the following formula:

FCR = Input of feed/Weight gained by the animal.

### 2.9. Data on Carcass Components

Two hens per replication were chosen at the ending of the experimental period; those BWG were closest to their subgroups' mean and maintained in a separate pen with no diet. So, at the end of experiment, the chicks were starved overnight, and they were individually weighed (to determine slaughter weight) and decimated. After de-feathering and removing the feet, skull, and internal organs, the dressed carcass weight was calculated, with the skin retained. The carcass yields, drumsticks, thighs, and breast were all prepared and weighted. The wings were removed through an upper limbs incision at the distal end of the tibia. It was possible to acquire the breast part. The thighs and drumstick parts were obtained by cutting throughout the junction between the femur and the ilium bone fragments of the coccyx. An incision across the junction made by the fibula, femur, and tibia severed that the drumstick from the thigh. The dressing % was estimated by dividing the dressed carcass weight by the slaughter weight.

RETRACTED

### 2.10. Blood Constituents Analysis

Analyses of proximate nutrients were performed through blood chemistry analysis by following way. For hematology constituents analysis, after the 1st experimental week (25-day-old chicks) and the last 5th experimental week (56-day-old chicks), the sample of blood were gathered from the wing's veins of two birds and were selected from each treatment in random way. Five milliliter (5 ml) blood was taken from the wing's a bird per treatment for hematology analysis. Samples of blood were taken in vials with anticoagulant two times during experimental period with each replicates. A complete blood count (CBC) test from the Kot Chutha medical lab in D. G Khan was used to calculate hematological components including RBC (red blood cell), WBC (white blood cell), HBG (hemoglobin concentration), MCHC (mean corpuscular hemoglobin concentration), MCH (mean corpuscular hemoglobin), GRA (granulocytes), PCV (pack cell volume), and MPV (mean platelet volume).

### 2.11. Statistical Analysis

The average feed consumption (intake) (g), average body weight and BWG (g), CBC, and output of carcass components were all analyzed using SAS software's one-way ANOVA. The means had compared by using DMR (Duncan multiple range) test. The results of the experimental trial were reported as mean ± standard error of the mean (SEM).

## 3. Results and Discussion

In this current study, the initial weight of the broilers (4 days old) chicks was not significantly different from each other, which shown that all the birds had uniform body weight at the start of experiment. After the acclimation periods of 21 days, the broiler chicks show uniform body weight at the age of 25 days and agreed with work of Fitasari and Mushollaeni [19] who report that body weight and feed intake show nonsignificant difference in commercial feeding during acclimation period until the age of 14 days which means that the impact of diet was not observed in the chicks during the commercial feedings.

### 3.1. Average Body Weight and Body Weight Gain (BWG)

The average body weight and BWG mean body weight gain are significantly different (*P* < 0.01) among the dietary treatments described in Tables 2 and 3. The broilers of treatment (*T*_2_) fed on (25% VW+75%) BF showed the highest final body weight and weight gain (*P* < 0.01) followed by other treatments that fed on the control treatment (*T*_1_) (0% VW+ 100%BF) and treatments (*T*_3_) (50% VW+ 50% BF) and (*T*_4_) (75% VW+25%BF), respectively, but not significantly different from control treatment (*T*_1_). In the diet of the broilers, the percentage of volume weight (VW) increased and resulted in less nutritional intake and stop the growth [20, 21]. Also the amount of the fiber increase in the diet resulted in poor nutritional value and feed efficiency [22]. The results of this study were fully agreed with the study of Oun [23] who reported that by the use of 25% VW in the diet of the broiler chicks, the FBW (final body weight) increased as compared to the diet of control treatment.

RETRACTED

### 3.2. Feed Intake and Feed Conversion Ratio (FCR)

In the current study, there was no significant effect (*P* > 0.05) on feed intake, but FCR was nonsignificant (*P* > 0.05) at the start and became significant at the end of experimental period (*P* < 0.05) as described in Tables 4 and 5 in accordance with Sakib et al. [24]; there was feed conversion ratio decreased at increased level of potato meal in broiler diet because the potato meal did not directly effect on the feed intake and growth performance of broiler chicks at 21, 28, 35, and 42 days of age. Maung et al. [25] observed that there was no significance difference (*P* > 0.05) at FCR and feed intake and body weight gain and live weight of broilers fed at 0 g, 34.5 g, and 69 g green vegetable (water spinach) with BF which promote the growth performance of broilers among dietary treatments agreed with current study at FCR and feed intake (*P* > 0.05) and showed controversy at live weight and body weight gain (*P* < 0.01) of broiler chicks. This study agreed with the study of Okapanchi et al. [26] who reported that there was no significant difference (*P* > 0.05) on feed intake of broilers on yam peels. He also observed that the amount of the fibers increases in the diet increases the feed intake in broiler chickens; the FCR did not show significant difference across the dietary treatments.

### 3.3. Carcass Components

Chicks fed on control diet (*T*_1_) had higher weight of the liver, dress carcass, breast meat, and drum stick weight than other dietary treatments which were significantly different (*P* < 0.05) from each other. But the lungs and large intestine are nonsignificant (*P* > 0.05) among different dietary treatments described in Table 6. This study agreed with the result of Melesse et al. [27] who observed the broilers who fed on (*T*_2_) (30 g/kg SPLM) had higher slaughter weight and things weight. The current study shows controversy with Mozafari et al.'s [28] work who used the different level of cooked and raw potato replacing with 25 and 35% seed of maize which reported that the dietary treatments had nonsignificant effect (*P* > 0.05) on weight of thighs, breast, and liver of broiler chicks.

RETRACTED

This study agreed with the results of Tamir and Tsega [29] who used the dried level of SPLM (sweet potato meal) at 0, 50, 100, 150, and 200 g/kg level which showed that drumstick, breast meat, and thighs are not affected with the dietary supplements because that material did not contain any dangerous effect on the health status and performance of the broiler chickens. The giblets' weight and the slaughter weight of broilers decrease with the increase of the supplemented feed as 100 g/kg dried sweet potato meal had gave higher giblets weight than 150 g/kg and 200 g/kg dried sweet potato meal.

### 3.4. Blood Constituents

The blood constituents in this study showed that broilers in all treatment groups fed on different doses were significantly (*P* < 0.05) different from each other. The value of RBC was lower in *W*_5_, and all other contents were higher in *W*_5_. The treatment (*T*_4_) had higher values of WBC, MID, GRA, HGB, MCV, and MPV in *W*_5_ than *W*_1_ that were significantly (*P* < 0.05) different from each other as described in Table 7. This study of blood constituent's controversy with the report of waken Elle (2010), who observed that in all the treatments, the values of the hemoglobin, RBC, and MCHC obtained were within the normal range. So, the highest values can be shown in hematocrit and mean corpuscular volume, and the mean corpuscular concentration was lower. This study show controversy with the study of [11] he used VW as 0%, 25%, 50%, 75% and 100% who reported that there was no significant difference in the immune status of broilers fed on different doses in different dietary treatments that decrease the intake of commercial by fed on more concentration of vegetable waste that not impact on the immune status of the broilers chicks. This study showed similarity at some extent with [30] who used 0%, 5%, 10%, and 15% Irish potato peel meal (IPPM) replaced with the maize in diet and observed that the blood constituents were significantly different (*P* < 0.05) from each other in different dietary treatments. The white blood cells were higher in control treatment (*T*_1_) but also similar with (*T*_4_) than (*T*_2_) and (*T*_3_) which were significantly different (*P* < 0.05). This study is in accordance with the report of [17] who reported that the concentration of HGB increased with the age of broilers.

## 4. Mortality

In the current study, there were no difference in the mortality of broilers during experimental periods agreed with the [19] work shown mortality on livestock experimental period experienced by illness or death in broiler chicks. The results of this study was also accordance with work of Whittemore et al. [31] and Agwunobi [32–36] who reported that the dietary treatments using potato did not show any significant effect (*P* > 0.05) on the mortality.

RETRACTED

## 5. Conclusion

Spinach, potato, and cauliflowers are the vegetables that have not enhanced and bettered the nutritional rate of the meat but also improved the color quality and taste of the meat of broiler chicks. In the current research, it is concluded that the dietary supplementation of vegetable waste had good effect on growth performance at 25% concentration in dietary treatment (*T*_2_). Consequently, appropriate and organized handlings of food waste (FW) not only produce the useful and energetic products but also minimize the crush on the environment. Processing food waste provides the valuable high nutritional organic part of food which would be reused for the animals as due to their nutritional values especially as for livestock food part.

## Figures and Tables

**Table 1:** Experimental design of feeding trials.

Dietary treatments	Inclusion rate of VW	Replications			
		*R*_1_	*R*_2_	*R*_3_	Total
*T*_1_ (control)	(0% VW+100% BF)	15	15	15	45
*T*_2_	(25% VW+75% BF)	15	15	15	45
*T*_3_	(50% VW+50% BF)	15	15	15	45
*T*_4_	75% VW+25% BF)	15	15	15	45
Total broiler chicks		60	60	60	180

**Table 2:** Average body weight for broiler chicks fed with different levels of VW (mean ± SEM).

Average body weight						
	Control: *T*_1_	*T*_2_	*T*_3_	*T*_4_	*P* value	Significance
Week 1	315 ± 0.86^b^	335.5 ± 0.86^a^	304.334 ± 0.61^c^	286.8334 ± 0.72^d^	.9071	NS
Week 2	567.5 ± 0.28^b^	585.83 ± 0.88^a^	548.167 ± 0.73^c^	503 ± 0.764^d^	.1939	NS
Week 3	872.67 ± 0.61^b^	898.667 ± 0.61^a^	863.5 ± 0.87^c^	836.334 ± 0.88^d^	.1233	NS
Week 4	1092.334 ± 0.44^b^	1115.167 ± 0.44^a^	1073.67 ± 0.601^c^	1042.834 ± 0.73^d^	.4274	NS
Week 5	1414 ± 0.76^b^	1507.167 ± 0.44^a^	1291 ± 1.041^c^	1256.167 ± 0.73^d^	.0184	^∗^

abc = means with same superscripts are non significant; ^∗∗^ = significant.

**Table 3:** BWG for broiler chicks fed with different levels of VW (mean ± SEM) during.

Body weight gain (BWG)						
	Control: *T*_1_	*T*_2_	*T*_3_	*T*_4_	*P* value	Significance
Week 1	207.5 ± 0.86^b^	226.5 ± 0.86^a^	196.34 ± 0.61^c^	180.834 ± 0.72^d^	.9071	NS
Week 2	460 ± 0.288^b^	476.83 ± 0.88^a^	440.167 ± 0.7^c^	397 ± 0.7637^d^	.1939	NS
Week 3	765.167 ± 0.6^b^	789.67 ± 0.61^a^	755.5 ± 0.86^c^	730.334 ± 0.88^d^	.1233	NS
Week 4	984.83 ± 0.44^b^	1006.167 ± 0.4^a^	965.667 ± 0.6^c^	936.834 ± 0.726^d^	.4274	NS
Week 5	1306.5 ± 0.76^b^	1398.167 ± 0.4^a^	1183 ± 1.041^c^	1150.167 ± 0.73^d^	.0184	^∗^

abc = means with different superscripts show that values are significantly different;^∗∗^ = significant.

RETRACTED

**Table 4:** Feed intake for broiler chicks fed with different levels of VW (mean ± SEM).

Feed intake						
	Control: *T*_1_	*T*_2_	*T*_3_	*T*_4_	*P* value	Significance
Week 1	617 ± 150.32	541 ± 4.583	450.667 ± 23.49	401.334 ± 22.06	.2751	NS
Week 2	776.67 *s* ± 49.16	1012.334 ± 111.78	816.334 ± 20.17	869 ± 78.71	.1966	NS
Week 3	1332.34 ± 56.37	1794.67 ± 197.12	1424 ± 93.724	1923 ± 298.61	.1519	NS
Week 4	2365.34 ± 173.28	2726.334 ± 289.60	2432 ± 393.85	2857.667 ± 07.26	.5740	NS
Week 5	3980 ± 107.59	4579 ± 62.978	4287 ± 240.251	4486.667 ± 242.66	.1750	NS

NS: nonsignificant.

**Table 5:** FCR for broiler chicks fed with different levels of VW (mean ± SEM).

Feed conversion ratio (FCR)						
	Control: *T*_1_	*T*_2_	*T*_3_	*T*_4_	*P* value	Significance
Week 1	2.1634 ± 0.0837	2.2167 ± 0.158	2.2934 ± 0.122	2.2134 ± 0.129	.9071	NS
Week 2	1.6834 ± 0.11	2.1167 ± 0.23	1.85 ± 0.045	2.1834 ± 0.202	.1939	NS
Week 3	1.7367 ± 0.074b	2.267 ± 0.24	1.88 ± 0.123	2.63 ± 0.407	.1233	NS
Week 4	2.38 ± 0.161a	2.7067 ± 0.29	2.51 ± 0.408	3.0467 ± 0.22	.4274	NS
Week 5	3.04 ± 0.08c	3.27 ± 0.046^bc^	3.59 ± 0.196^ab^	3.897 ± 0.212^a^	.0184	^∗^

NS: nonsignificant.

**Table 6:** Carcass components weight of broiler chicks fed with different levels of VW (mean ± SEM).

Carcass components						
	Control: *T*_1_	*T*_2_	*T*_3_	*T*_4_	*P* value	Significance
Slaughter weight (g)	1413.167 ± 0.7^b^	1506.5 ± 0.5^a^	1290.167 ± 1.01^c^	1255.34 ± 0.60^d^	.9071	NS
Dress carcass (g)	901 ± 2.08^a^	881.34 ± 1.8^b^	863.67 ± 0.8^c^	802.334 ± 1.45^d^	.1939	NS
Dressed %	63.734 ± 0.12^b^	58.476 ± 0.107^c^	66.89 ± 0.03^a^	63.537 ± 0.26^c^	.1233	NS
Breast meat %	28.71 ± 0.12^a^	26.72 ± 0.12^b^	22.17 ± 0.04^c^	20.101 ± 0.17^d^	.4274	NS
Thighs %	13.23 ± 0.036^d^	19.51 ± 0.04^a^	16.92 ± 0.109^b^	16.4584 ± 0.09^c^	.0184	^∗^
Drum stick (%)	12.54 ± 0.089^a^	16.561 ± 0.09^b^	15.821 ± 0.14^b^	15.4853 ± 0.06^c^	.9071	NS
Wings (%)	11.5203 ± 0.16^d^	13.002 ± 0.136^b^	12.33 ± 0.09^c^	14.68 ± 0.165^a^	0.011	^∗∗^
Gizzard (%)	2.976 ± 0.015^c^	4.97 ± 0.08^a^	4.667 ± 0.08^a^	4.337 ± 0.14^b^	0.013	^∗∗^
Liver (%)	3.4944 ± 0.05^a^	3.239 ± 0.04^b^	1.99 ± 0.018^d^	2.388 ± 0.03^c^	0.015	^∗∗^
Heart (%)	0.65 ± 0.012^d^	0.803 ± 0.04^c^	0.9708 ± 0.028^b^	1.185*b* ± 0.03^a^	0.017	^∗∗^
Lungs (%)	0.703 ± 0.018^a^	1.045 ± 0.013^a^	0.798 ± 0.39^a^	0.821 ± 0.0254^a^	0.673	NS
Kidney (%)	0.607 ± 0.018^d^	0.86 ± 0.029^c^	1.009 ± 0.019^b^	1.18767 ± 0.02^a^	0.013	^∗∗^
Small intestine (%)	7.117 ± 0.038^d^	7.46 ± 0.013^c^	7.84 ± 0.031^b^	8.82134 ± 0.04^a^	0.014	^∗∗^
Large intestine (%)	0.86 ± 0.0145^a^	0.857 ± 0.37^a^	0.89 ± 0.032^a^	0.595 ± 0.043^a^	0.662	NS

abc = means with different superscripts on the different rows among the different treatments are significantly different;^∗∗^ = significant; NS: nonsignificant.

RETRACTED

**Table 7:** Blood constituents for broiler chicks fed with different levels of VW (mean ± SEM).

Blood constituents						
	*T*_1_	*T*_2_	*T*_3_	*T*_4_	*P* value	Significance
WBC (10^3/uL)	110.26 ± 1.56^c^	121.97 ± 1.90^a^	105.29 ± 5.2^d^	115.72 ± 8.525^b^	.9071	NS
LYM (10^3/uL)	99.04 ± 0.92^b^	109.22 ± 0.52^a^	92.97 ± 1.95^c^	98.68 ± 3.77^b^	.1939	NS
MID (10^3/uL)	7.88 ± 0.918^c^	8.93 ± 0.747^b^	7.58 ± 1.298^c^	13.11 ± 3.556^a^	.1233	NS
GRA (10^3/uL)	3.75 ± 1.53^d^	3.80 ± 1.487^c^	4.60 ± 1.889^b^	7.80 ± 3.338^a^	.4274	NS
RBC (10^6/uL)	2.17 ± 0.023^b^	2.30 ± 0.008^a^	1.95 ± 0.090^c^	1.46 ± 0.174^d^	.0184	^∗^
HGB (g/dL)	9.15 ± 0.086^a^	9.08 ± 0.048^a^	7.85 ± 0.45^c^	8.65 ± 0.52^b^	.9071	NS
MCHC (g/dL)	33.99 ± 0.08^b^	34.17 ± 0.62^b^	34.58 ± 0.85^b^	50.67 ± 6.32^a^	.1939	NS
MCH (pg)	42.07 ± 0.574^b^	39.72 ± 0.236^c^	39.53 ± 0.65c	66.20 ± 11.449^a^	.1233	NS
MCV (fL)	124.48 ± 1.38^b^	117.68 ± 3.09^d^	118.67 ± 3.73^c^	125.43 ± 7.08^a^	.4274	NS
MPV (fL)	3.72 ± 0.06^b^	3.68 ± 0.09^b^	3.68 ± 0.083^b^	4.20 ± 0.23^a^	.0184	^∗^

abc = means with different superscripts on the same rows among the different treatments are significantly different;^∗∗^ = significant.

## Data Availability

All data is available within the manuscript.
